# Abnormal Target Detection Method in Hyperspectral Remote Sensing Image Based on Convolution Neural Network

**DOI:** 10.1155/2022/9223552

**Published:** 2022-05-17

**Authors:** Yun Liu, Jia-Bao Liu

**Affiliations:** ^1^School of Information Engineering, Chaohu University, Chaohu 238024, China; ^2^School of Mathematics and Physics, Anhui Jianzhu University, Hefei 230601, China

## Abstract

Abnormal target detection in hyperspectral remote sensing image is one of the hotspots in image research. The image noise generated in the detection process will lead to the decline of the quality of hyperspectral remote sensing image. In view of this, this paper proposes an abnormal target detection method of hyperspectral remote sensing image based on the convolution neural network. Firstly, the deep residual learning network model has been used to remove the noise in hyperspectral remote sensing image. Secondly, the spatial and spectral features of hyperspectral remote sensing images were used to optimize the clustering dictionary, and then the image segmentation containing target information is completed. Finally, the image was input into the deep convolution neural network with a dual classifier, and the network detects the abnormal target in the image. The test results of this algorithm show that the structural similarity of the denoised image is higher than 0.86, which shows that this method has good noise reduction performance, image details will not damage, segmentation effect is good, and it can obtain high-definition target image information and accurately detect abnormal targets in the image.

## 1. Introduction 

Remote sensing images, also known as remote sensing images, include aerial photos and satellite photos. Therefore, the imaging methods of remote sensing images include aerial photography, scanning, or microwave radar scanning [1]. With the continuous development of remote sensing technology, the requirements for the imaging effect and quality of remote sensing images are gradually improved, from the basic monitoring application to the detection of abnormal targets through remote sensing images. Therefore, the resolution of remote sensing images needs to reach a certain standard. Based on this, hyperspectral is applied in the field of remote sensing and combined with remote sensing technology to obtain hyperspectral remote sensing images with better resolution [2]. Hyperspectral image refers to the resolution of 10–2*λ* for images of orders of magnitude, and spectral sensors are deployed on different space platforms to image the target area [3], which can obtain its surface image and spectral image at the same time, to realize the combination of spectrum and remote sensing. The convolution neural network is a kind of network with the ability of convolution calculation and representation learning. It is widely used in image and object recognition, pose estimation, natural language processing, and so on. Moreover, the network has a good effect in processing the geometric, texture, and spatial distribution characteristics of remote sensing images and can identify the target objects in remote sensing images. In order to realize the detection of abnormal targets in hyperspectral remote sensing images [4], after relevant research in the literature [5] and [6], a correlation detection method based on spatial spectrum joint anomaly degree and spectral difference equalization interval screening is proposed. In the detection process, the above method has no segmentation effect and cannot accurately obtain the target area information. Therefore, there is a certain error in the detection result of the above method. Therefore, this paper proposes an abnormal target detection method of hyperspectral remote sensing image based on the convolution neural network. Firstly, the high-frequency layer with noise information is studied in multiscale space by the residual network, and the residual remote sensing image is generated by residual mapping. Finally, the complete denoising result is obtained by jump connection. Then, the dictionary learning model is used to obtain the sparse representation of the brightness component and color image of the remote sensing image, reconstruct and compensate the missing high-frequency information in the remote sensing image, retain the high-resolution of the image, and retain the spectral information and spatial detail information in the remote sensing image. Finally, the convolution neural network is used to segment the hyperspectral remote sensing image after extracting the features and finally complete the image abnormal target detection.

## 2. Detection of Abnormal Targets in Hyperspectral Remote Sensing Images

### 2.1. Denoising of Hyperspectral Remote Sensing Image Based on Depth Residual Learning

In the process of imaging acquisition of hyperspectral, remote sensing images, under the influence of environment, equipment, and other factors, there will be noise in the acquired images, which will affect the detection results [7]. Therefore, in order to ensure the accuracy of abnormal target detection in hyperspectral remote sensing images, this paper uses depth residual learning to denoised the images.

Deep residual learning is a deep network model including residual module, which is composed of residual units. There is a mapping relationship between hyperspectral remote sensing images before and after noise reduction, which is nonlinear. The mapping relationship is realized by inputting the high-frequency band noise data in the image into the residual module technology. Multiple data nodes are connected by jumping, and each module can be effectively connected, so as to retain more edge information in the semantic feature difference information. The core of the network is the residual of the connection depth (shortcut connections), introducing branches to ensure smooth network data transmission and avoid under fitting caused by gradient disappearance and degradation.

#### 2.1.1. Input Layer

The original hyperspectral remote sensing image *y* (*x*) is used as the input of the model and input by the input layer.

#### 2.1.2. Feature Extraction Layer

This layer completes the feature extraction of hyperspectral remote sensing image in the form of image block. In this process, the feature is extracted to ensure that the image features will not change after noise reduction. Map the image block originally located in the image space to the feature space, complete the learning of image features, and take the feature as a filter to participate in the convolution operation of the original hyperspectral remote sensing image. Its purpose is to obtain the activation value, which belongs to different positions and features of the original image. In this layer, the activation function and convolution kernel are used to extract the eigenvalues of the image block, and the obtained neurons are transmitted to the residual module.

#### 2.1.3. Residual Module

It mainly completes the residual learning between the input and output of the whole model. In order to ensure the integrity of image detail information in the learning process, this paper introduces local residual learning and recursive block and adjusts the residual module so that the input of identity branch and residual branch are in two states in the model and recursive block. The former is difference, and the latter is the same. In this way, the path between the input and output of recursive block is multipath, which can effectively avoid the phenomenon of overfitting. To improve the learning performance of the model, formula (1) of the residual unit is as follows:

(1) $$\begin{array}{c} H^{u}=g\left(H^{u-1}\right)=\left(F_{H^{u-1}},F_{W}\right)+H^{0}, \end{array}$$

where *g* represents the function, corresponding to the residual unit; *F*_*W*_ represents residual function; and both *H*^0^ and *H*^*u*^ represent the output. The former corresponds to the first convolution layer, and the latter corresponds to the residual unit; *F*_*H*^*u*−1^_ is the input of the unit; *u* represents quantity, corresponding to residual unit. The original expectation mapping skips one or more layers of network structure and realizes identity mapping. With the increase of network depth, the weight of the convolution layer is constantly updated, and the weight value iterates in the direction of gradient descent.

#### 2.1.4. Network Reconstruction Layer

After learning, the residual unit outputs the characteristic map of the image block and transmits it to this layer to form a hyperspectral mapping image, and its number is the same as the original image. After fusion processing through convolution calculation, a complete hyperspectral remote sensing image is formed. This layer can complete the prediction and removal of noise components in the image [8], so as to obtain the denoised hyperspectral remote sensing image. Then, the calculation formula is as follows:

(2) $$\begin{array}{c} X_{x}=x\times \left(H^{u}-s\right), \end{array}$$

where *x* represents the image after noise reduction; *X*_*x*_ represents the residual noise image after residual learning. The network learns the mapping from noise image to noise distribution. Using the characteristics of the neural network and global jump connection, *x* is subtracted to obtain a complete denoised image, and the multiplicative noise is removed indirectly by subtraction.

### 2.2. Feature Extraction of Hyperspectral Remote Sensing Image

In the abnormal target detection of hyperspectral remote sensing image, it is necessary to accurately extract the target information in the image. Therefore, this paper guarantees the definition of remote sensing image on the basis of noise reduction and then carries out feature segmentation on *x* to remove the background in the image and retain the feature information. This paper uses the clustering dictionary learning method combined with the residual network model to complete the image pixel segmentation.

Determine the cluster center, use the dictionary representation, determine the category attribution, and complete the dictionary learning, which are completed according to the sparse representation and the elements in the cluster, respectively. In order to better characterize the image features [9], the dictionary atom is described based on the region image block. The dictionary is optimized by combining the two characteristics of wide band range and high-spectral resolution of hyperspectral remote sensing image, and the segmentation is completed by using the optimized DICTIONARY [10].

The purpose of clustering is to realize the division of clusters, which is completed according to the similarity of images, so that the elements with increased similarity are located in the same cluster, as shown in the following formula:

(3) $$\begin{array}{c} W_{a}=\min\sum_{i=1}^{K}R\left(x_{i},\upsilon_{i}\right), \end{array}$$

where *K* represents the number of clusters; *x*_*i*_ represents the *i* cluster, and *v*_*i*_ represents its cluster center; *R* represents the input hyperspectral remote sensing image, and *R*(*x*_*i*_, *v*_*i*_) represents the distance, corresponding to the distance between *x*_*i*_ and *v*_*i*_. The smaller the distance, the higher the degree of similarity between the two.

*x*_*j*_ is classified according to *V*_*i*_. On this basis, a new clustering center is obtained, and the clustering is completed after complete convergence through cyclic iterative processing between them.

The center point is determined and represented by any pixel in *x*_*j*_. In order to obtain the column vector set and contain *n* elements, the neighborhood image is processed by transformation, and the set is used as the input signal. The objective function of the method is shown in formula (1):

(4) $$\begin{array}{c} \underset{w_{ij},D_{j},C_{j}}{\min}J=\underset{w_{ij},D_{j},C_{j}}{\min}\sum_{j=1}^{k}\sum_{x_{i}\in C_{j}}\left(x_{i}-D_{j}w_{ij}\right), \end{array}$$

where *k* represents the limit; *J* represents the sparse vector value; C_*j*_ represents the number of atoms; *D*_*j*_ stands for dictionary, corresponding to *C*_*j*_; *m*_*j*_ represents the number of atoms, corresponding to *D*_*j*_; *w*_*ij*_ represents sparse vector, corresponding to any signal *x*_*i*_; *T* represents the limit, corresponding to sparsity; *R*(*D*_*j*_) represents the function, which is used to judge the consistency within *D*_*j*_; *δ* means to set the fluctuation threshold. The smaller the value, the higher the consistency of atoms in the dictionary.

After completing the construction of *D*_*j*_, each *w*_*ij*_ has corresponding pixels in different clustering dictionaries. Therefore, the former can be determined according to the image signal corresponding to the latter. If you get ‖*x*_*i*_ − *D*_*j*_*w*_*ij*_‖ with the smallest *D*_*j*_, it indicates that the similarity between *D*_*j*_ and *x*_*i*_ is high, you can classify the latter into the former.

During image segmentation [11], the neighborhood information of each pixel of hyperspectral remote sensing image is processed by transformation to form a one-dimensional vector *x*_*i*_. In order to obtain the input signal set *X*, all signals are integrated to obtain *x*_*i*_, which belongs to spectral remote sensing image. After the sparse representation of *X* is completed by sparse coding, *X*_*i*_ is segmented by clustering. In order to ensure the matching degree between the dictionary and the signal, the dictionary update needs to be completed, which is completed according to the signal in the cluster. After realizing the convergence of the energy function value *J* according to the cyclic interactive iteration, the clustering segmentation of hyperspectral remote sensing image is completed, and the segmented image $\tilde{X}$ containing target information is obtained.

### 2.3. Abnormal Target Detection Based on Deep Convolution Neural Network

After image clustering and segmentation, this paper uses the deep convolution neural network (DCNN) model to complete the final hyperspectral remote sensing image abnormal target detection. The model adopts dual classifier. The classifier is a machine learning method based on quadric surface and a general abnormal target linear classification method. Thus, the final abnormal target detection is completed, and the model structure is shown in Figure 1.

Take $\tilde{X}$ as the input of the model, and the convolution layer extracts the feature of $\tilde{X}$. Through convolution operation, the feature signal of the image can be enhanced, and the edge detection of the image can be sharpened and blurred [12]. The formula of convolution operation process is shown in

(5) $$\begin{array}{c} a_{j,l}=f\sum_{i\in M_{j}}\tilde{X}a_{j,l-1}*f\kappa_{i,j,l}fb_{j,l}, \end{array}$$

where *a*_*j*, l_ represents the activation value, corresponding to the output characteristic image *j*, and belongs to layer *l*; *k*_*i*, *j*, l_ represents the kernel, which is used to connect two characteristic diagrams, which are located in layer *l* and layer *l* – 1, respectively; *b*_*j*,l_ represents the addition deviation, which corresponds to the output characteristic image *j*, and belongs to layer *l*; *f*(·) represents Relu function; *M*_*j*_ represents the characteristic diagram *j* and is linear.

The pooling layer can realize subsampling processing, which belongs to image features and needs to be based on the local correlation of the image, so that the valuable information in the image can be retained to the greatest extent [13]. The calculation formula of this layer is

(6) $$\begin{array}{c} a_{j,l}=f\beta_{j,l}\text{down}\left(a_{j,l-1}\right)\tilde{X}+f\alpha_{j,l}b_{j,l}, \end{array}$$

where down(·) represents the function, corresponding to subsampling; *β*_*j*,1_ and *α*_*j*,1_ represent multiplication bias, corresponding to the output characteristic image, and belong to the layer *l*.

When detecting abnormal targets in hyperspectral remote sensing images [14], there are obvious quantitative differences between classes. Therefore, in order to ensure the accuracy of detection results, weight is introduced to restrict each class of the image, larger weight is added to smaller classes, and smaller weight is added to larger classes; then, as shown in the following formula,

(7) $$\begin{array}{c} L\left(W,b\right)=\frac{1}{2}\left[\frac{\sum_{i=1}^{z}\mu_{i}{\left\|y_{j}^{z_{i}}-{\overset{⌢}{y}}_{j}^{z_{i}}\right\|}^{2}}{mn}+\lambda W^{T}W\right], \end{array}$$

where *μ*_*i*_ represents the weight, which is used for different types of constraints; *L* represents the deformation of norm; *z*_*i*_ represents the quantity, corresponding to the selected hyperspectral remote sensing image sample points; *λ*, *m*, and *n* are constants; *W* represents the weight matrix; *y*_*j*_^*z*_*i*_^ and ${\hat{y}}_{j}^{z_{i}}$ represent the feature value and feature approximation of the selected image, respectively.

The dual classifier in the model is a two-layer stack. The first layer is used as the training set of the second layer after completing the feature reconstruction of hyperspectral remote sensing image [15]. The dual classifier has the ability of spectral remote sensing image feature fusion, which can fuse the original features and extracted new features in the image, and process the fused features by means of standardization and normalization, to improve the detection accuracy of abnormal targets.

## 3. Experimental Analysis

In order to test the application performance and effect of this method on the abnormal target detection of hyperspectral remote sensing image, this method is used to detect the remote sensing image of land resource management in a province. The purpose of detection is to determine the abnormal illegal construction or illegal occupation of cultivated land based on hyperspectral remote sensing image and cooperate with relevant departments to complete land resource management. Hyperspectral remote sensing image detection is used to collect abnormal information. In the process of real-time abnormal target detection, line images need to be collected, so a 2-way blade server is used as the image server. Considering the running time, a disk array with a capacity of 8 t will be selected for the amount of data collected, so as to ensure the safety of abnormal target detection in hyperspectral remote sensing images.

### 3.1. Denoising Test

In order to test the drying performance of this method, structural similarity *S*_SSIM_(*x*, *y*), image information entropy *H*, and average correlation coefficient $\bar{C}$ are used as rating indicators, in which structural similarity refers to the measurement of macromolecular structural similarity; image information entropy refers to the average number of bits in the gray level set of hyperspectral remote sensing images; average correlation coefficient refers to the amount of linear correlation between abnormal target detection variables in hyperspectral remote sensing images, which usually represents an uncertain relationship. Test the results of three indexes after image denoising with different noise levels, as shown in Figures 2–4. The calculation formulas of the three indicators are as follows:

(8) $$\begin{array}{c} S_{\text{SSIM}}\left(x,y\right)=\frac{2\varepsilon_{x}\varepsilon_{y}}{{\left(\varepsilon_{x}+\varepsilon_{y}\right)}^{2}}\frac{2\sigma_{xy}}{{\left(\sigma_{x}+\sigma_{y}\right)}^{2}}, \end{array}$$

(9) $$\begin{array}{c} H=-\sum_{i=0}^{1}p{\left(i\right)}^{2}\ln, \end{array}$$

(10) $$\begin{array}{c} \bar{\vartheta }=\frac{\sum_{i=1}^{m}\sum_{j=1}^{n}\vartheta_{o\;d}\left(i,j\right)}{mn}, \end{array}$$

where *x* and *y* represent two hyperspectral remote sensing images, and their mean values are represented by *ε*_*x*_ and *ε*_*y*_, respectively. The covariance between them is *σ*_*xy*_; *P*(*i*) represents the probability density function, corresponding to the gray value *i*. *ϑ*(*i*, *j*) represents the correlation coefficient, which belongs to the spectral vector before and after noise reduction and corresponds to the pixel at (*i*, *j*) of the hyperspectral remote sensing image; *m*, *n* represent the number of rows and columns of hyperspectral data, respectively. The larger the value of the three index results, the better the noise reduction performance of this method, and the more the details and quality of the denoised image can be guaranteed. The expected standard is that the results of the three indexes are higher than 0.86.

According to the test results of Figures 2–4, under different image sizes, with the gradual increase of noise, the three indicators of this method show corresponding differential changes, but the change results meet the expected standard requirements, even if the image size is 80 × 80, when the noise is 20 dB, the results of the three indexes are 0.91, 0.90, and 0.88, respectively. Therefore, this method has good noise reduction performance.

In order to measure the noise reduction effect of this method, a remote sensing image of land resource management is randomly selected for noise reduction and the image results before and after noise reduction are obtained to judge the noise reduction effect of this method, as shown in Figure 5.

### 3.2. Image Classification and Evaluation

In the experiment of remote sensing image classification, this paper uses 2DCNN, 3DCNN, and ResNet to compare and analyze the classical Indian pins set of remote sensing data, so as to further verify the training advantages of residual network. As shown in Table 1, the OA of remote sensing image classification completed by the reset model is as follows: the value is 0.966385; the value of AA is 0.967972; and the value of kappa is 0.960746.

Figure 6 shows the confusion matrix of the classification of Indian pins common data set. It is found that the position of each measured pixel shows better accuracy compared with the corresponding position of the actual image.  Figure 7 shows the iterative values of loss, accuracy, val_loss, and val_loss, which further shows that this method has a good effect on the classification of multiband remote sensing images after noise removal.

According to the test results in Figures 5–7, it can be seen that there is noise influence in the image before noise reduction, and there is fuzziness in the image. After noise reduction, the clarity and brightness of the image are significantly improved. The results intuitively show that the noise reduction effect of this method is good, and the noise removal in the image can be completed on the premise of ensuring the quality of image details.

In order to test the image segmentation effect of the method in this paper, the gray mean and Jaccard similarity are used as evaluation indexes, and their calculation formulas (11)-(12) are as follows:

(11) $$\begin{array}{c} \mu =\frac{1}{mn}\sum_{i=1}^{m}\sum_{j=1}^{n}x_{ij}, \end{array}$$

(12) $$\begin{array}{c} \text{JAC}\left(A,B\right)=\frac{\left|A\cap B\right|}{\left|A\cup B\right|}, \end{array}$$

where *x*_*ij*_ represents the gray value of the image after noise reduction and corresponds to the pixel point at (*i*, *j*); *A*, *B* represent two different sets. The average gray level can reflect the gray level of the image, that is, the brightness of the image, and the expected standard is between 0.4 and 0.6. The closer the JAC similarity is to 1, the better the quality of the segmented image. The expected standard in this paper is more than 0.85.

The image segmentation results of the method in this paper are obtained according to formulas (9) and (10), as shown in Figures 8 and 9.

According to the test results of Figures 8 and 9, with the gradual increase of the number of segmentation of hyperspectral remote sensing images, the results of gray mean fluctuate within the standard range. The results show that even if the number of segmentation is large, the basis can ensure the image quality. Therefore, it also indirectly shows that. The segmentation effect of this method is still good for images with complex background. In addition, with the gradual increase of clustering centers in the image, the results of JAC similarity fluctuate irregularly, but the variation range is about 0.9. Therefore, the image segmentation effect of this method is good and can obtain the target image information with high definition.

### 3.3. Target Monitoring Results

In order to test the abnormal target detection of hyperspectral remote sensing image in this method, this method is used to detect the abnormal target in the denoised image in Figure 5. There are abnormal illegal buildings in this image. The detection results of this method are obtained, as shown in Figure 10.

According to the test results in Figure 10, this method can complete the detection of abnormal targets in hyperspectral remote sensing images and obtain abnormal illegal buildings in the images. After confirmation, the detection results are consistent with the actual results. Therefore, this method has the effect of abnormal target detection in hyperspectral remote sensing images, and the detection results have good reliability.

## 4. Conclusion

Hyperspectral remote sensing images are used in more and more fields. It is an important detection method to complete abnormal target detection based on remote sensing images. In order to ensure the reliability of hyperspectral remote sensing image abnormal target detection, a hyperspectral remote sensing image abnormal target detection method based on the convolution neural network is proposed in this paper. The convolution neural network is used to classify the image to obtain the high-spectrum remote sensing image with target features, which is introduced into the convolution neural network with dual classifier to detect it. The results show that the abnormal target detection method of hyperspectral remote sensing image based on the convolution neural network has good noise reduction performance and can complete the noise processing in the image under the condition of ensuring the image quality and fine grain level. At the same time, it can also better complete the classification of target areas, and the display effect of various indicators is good. After segmentation, the quality of hyperspectral remote sensing image is intact, which plays an important role in accurately detecting abnormal targets in the image.

## Figures and Tables

**Figure 1:** Abnormal target detection model based on DCNN hyperspectral remote sensing image.

**Figure 2:** Test results of the structural similarity index.

**Figure 3:** Test results of the image information entropy index.

**Figure 4:** Test results of the average correlation coefficient index.

**Figure 5:** Test results of noise reduction effect.

**Figure 6:** Confusion matrix of the residual network.

**Figure 7:** Precision contrast of the residual network.

**Figure 8:** Test results of the gray mean index.

**Figure 9:** JAC similarity index test results.

**Figure 10:** Abnormal target detection test results.

**Table 1:** Comparison of classification accuracy of remote sensing images.

Network type classification criteria	OA	AA	Kappa
2DCNN	0.761929	0.767287	0.728459
3DCNN	0.949264	0.970596	0.940559
ResNet	0.966385	0.967972	0.960746

## Data Availability

The datasets generated for this study are included within the article.
